# Scaling Human-Object Interaction Recognition in the Video through Zero-Shot Learning

**DOI:** 10.1155/2021/9922697

**Published:** 2021-06-09

**Authors:** Vali Ollah Maraghi, Karim Faez

**Affiliations:** Department of Electrical Engineering, Amirkabir University of Technology (Tehran Polytechnic), Tehran, Iran

## Abstract

Recognition of human activities is an essential field in computer vision. The most human activity consists of the interaction between humans and objects. Many successful works have been done on human-object interaction (HOI) recognition and achieved acceptable results in recent years. Still, they are fully supervised and need to train labeled data for all HOIs. Due to the enormous space of human-object interactions, listing and providing the training data for all possible categories is costly and impractical. We propose an approach for scaling human-object interaction recognition in video data through the zero-shot learning technique to solve this problem. Our method recognizes a verb and an object from the video and makes an HOI class. Recognition of the verbs and objects instead of HOIs allows identifying a new combination of verbs and objects. So, a new HOI class can be identified, which is not seen by the recognizer system. We introduce a neural network architecture that can understand and represent the video data. The proposed system learns verbs and objects from available training data at the training phase and can identify the verb-object pairs in a video at test time. So, the system can identify the HOI class with different combinations of objects and verbs. Also, we propose to use lateral information for combining the verbs and the objects to make valid verb-object pairs. It helps to prevent the detection of rare and probably wrong HOIs. The lateral information comes from word embedding techniques. Furthermore, we propose a new feature aggregation method for aggregating extracted high-level features from video frames before feeding them to the classifier. We illustrate that this feature aggregation method is more effective for actions that include multiple subactions. We evaluated our system by recently introduced Charades challengeable dataset, which has lots of HOI categories in videos. We show that our proposed system can detect unseen HOI classes in addition to the acceptable recognition of seen types. Therefore, the number of classes identifiable by the system is greater than the number of classes used for training.

## 1. Introduction

Humans play a significant role in most of the activities that take place in the world. Human action recognition is one of the fundamental problems in computer vision and has many applications, such as video navigation, human-robot collaboration, and predicting human behavior for security purposes. Many human activities are made up of two parts: a verb and an object. The verb is what a man does on an object. In fact, a verb represents the movement of the human body. This type of activity is referred to as human-object interaction (HOI). For example, “opening the door” or “reading a book” has a verb and an object. Therefore, recognizing HOI is as important and challenging as recognizing human activities in the field of machine vision.

Many researchers have been working on human-object interaction (HOI) understanding [1–6]. HOI understanding can be followed in images or videos (sequence of frames). Distinguishing the full range of human activities in real environments is a significant challenge in computer vision. Some problems are as follows: large intraclass variation in actions, high variability in spatiotemporal scaling, human pose variations, occlusions, and, most importantly, the vast space of human activities. The most effective HOI recognition task methods are methods based on deep learning approaches that need a lot of labeled data [6–11]. The existing machine learning approaches for action understanding require fully annotated datasets. Some datasets have been prepared for this purpose, such as the “Humans Interacting with Common Objects” dataset for action classification (HICO) [3] and action detection (HICO-DET) [5] that are image benchmark. For HOI analysis in videos, not many datasets are provided. Charades dataset [12] was recently supplied for the HOI understanding tasks in video data. It has many human-object interaction categories and is suitable for action detection, HOI recognition, and video captioning purposes.

One of the essential HOI recognition challenges is the high number of possible categories in the real environment. Since the space of possible HOIs in real situations is enormous, list all possible HOI classes and obtain enough data for each group, and annotating the collected data is impractical. How can we reduce the need for training data for training an HOI recognizer model? Can a recognition model be taught with data from only part of the target classes? We focus on this question and tackle it through zero-shot learning for scaling HOI recognition in video data. In the recognition approaches based on zero-shot learning, the main class is decomposed into its components, and recognizing the main class components is applied instead of understanding the main category. So, the recognizer model learns the components of unseen classes that probably appear in other seen classes. In this case, if components of the novel HOI class appeared in other seen HOI classes, the model can recognize them and identify the new HOI class. Zero-shot learning for scaling HOI recognition is used previously for image data [13]. Our previous work presented a simple structure for zero-shot recognizing of HOI in video data [14].

In this work, we expand our previous work [14] and address the scaling of human-object interaction in video data through zero-shot learning. In this approach, the HOIs decompose into verbs and objects as the components of an HOI. For each input video containing an HOI, the detection system recognizes a verb and an object. For this purpose, the central proposed scheme has a two-branch deep neural network structure consisting of object recognition and verb recognition branches. A convolutional neural network (CNN) is used to extract the feature maps of each frame. We use recurrent neural networks (RNNs) in the verb recognition branch due to the video's temporal information. RNNs can represent the long dependencies in video data, which can help recognize verbs in the video.

We propose using lateral information to combine the verbs and the objects better to make valid verb-object pairs. It helps to prevent the detection of rare and probably wrong HOIs. The lateral information comes from word embedding techniques.

We also propose a new feature aggregation method for aggregating extracted high-level features from video frames before feeding them to the classifier. We use a local feature aggregation method that does not turn the entire extracted features space into a single space. We illustrate that this feature aggregation method is more effective for actions that include multi subactions.

We evaluate our proposed algorithm on the Charades dataset [12] and illustrate that our model can identify the novel HOI categories not seen by the model before. The Charades dataset has many human-object interaction categories and is suitable for action detection, HOI recognition, and video captioning purposes. This dataset contains 9848 video clips of HOIs captured in real environments. It has 157 categories of human activities, including some actions with “no interaction,” 149, which can be considered valid verb-object pairs. This 149 category consists of 34 verbs and 37 objects. Also, we compare our model in a fully supervised manner with the best-reported methods on this dataset and show that our method's performance can be comparable to them.

This study's primary purpose is to reduce the need for data to train an HOI recognition system by increasing the number of identifiable HOIs without increasing HOIs in training data. We focus on this purpose through zero-shot learning, in which we decompose the HOI into a verb (human action) and an object and recognize them in the video. We use CNNs and RNNs for implementing our proposed algorithm.

In the rest of the paper, we review some related works in part 2. The model architecture and proposed algorithm are presented in Section 3. We present the experimental results, evaluations, and discuss the results in Section 4, and conclude in Section 5.

## 2. Related Works

### 2.1. Human Action and HOI Recognition

Initial works on understanding human activities were in modeling actions. Many works can be found that used semantics for modeling and understanding of activities [15]. The HOI modeling started with the affordances idea introduced by J. Gibson [16], and then some works were done in the field of functionality understanding of objects and verbs [17]. Several approaches have been used to model semantic relationships [18, 19] for HOI understanding. Modeling humans and objects' spatial relationships using the interactional features are introduced by Delaitre et al. [20]. Also, learning distributed representations of humans and objects by poselet [21] and phraselets [22] are proposed for HOI recognition. Most of these efforts require costly-labeled data (pose, body parts, and object segmentation, etc.), making it difficult to collect data for any type of activity and make them applicable for cases with a limited number of classes. In fact, they fail for cases with more classes.

Recently, with providing large datasets [3, 5, 23] and the success of neural network-based approaches in classification and recognition tasks, the problem of understanding and recognizing HOIs has received a lot of attention. Inspired by this impressive progress, the researchers tried to develop deep networks for video analysis applications such as action recognition [24–28] and HOI understanding [23, 29].

The recognition in video is more complicated than recognition in still images because of the complexity of video sequences' motion patterns. Therefore, the mere use of appearance cues for successful recognition may not be enough. Most existing approaches have introduced a two-stream framework that considers both temporal and spatial domains [25, 30–37]. Classifiers operate on the two streams of inputs, the RGB and the optical flow, as spatial and temporal cues, respectively. Motion cues are used separately from appearance cues for final representing in the video. Two streams are trained individually in the training phase, and the outputs of them fuse to predict the output class in the testing phase.

Some approaches use 3D networks that work by spatiotemporal convolutions [26]. These networks usually consider a short video interval with a predefined number of frames and encode the local and short-term motion patterns. For example, 15, 7, 16, and 2 frames are used in [26, 30, 38, 39]. Also, other types of spatiotemporal networks like RNNs [26] and the extended versions of them which are called Long Short-Term Memory (LSTM) [40] are used to describe the temporal cues for video classification. The approaches based on spatiotemporal networks have a huge amount of computing due to many trainable parameters tuned in the training phase. A component-based approach is proposed to represent the video content, weakly supervised learning (WSL) method [41], and requires less annotated data. A three-stream CNN is suggested that receives two representations and were fused with the motion-encoding stream. The LSTM block models each of the three streams' temporal relationship. For the fusion of the three streams and the final prediction generation, an fc layer is used.

The literature study showed that the best methods for activity understanding are the deep learning-based approach. An essential issue in these methods is much data for all recognizable classes required for model training. They are only able to detect activities seen by the model. Providing the training data for all possible HOI categories is costly and impractical. We focus on this problem and try to solve it through the zero-shot learning approach.

### 2.2. Zero-Shot Learning

Zero-shot learning is an exciting approach in different areas [42–45]. Most new methods based on zero-shot learning have two stages and focus on attributes [46–50]. The attributes are predicted in the first step and then infers class labels in the second step. The compositional learning for Visual Question Answering (VQA) has been explored [51], in which the VQA task breaks down into a sequence of modular subproblems. Each subproblem is modeled by one neural network.

For zero-shot action recognition, simultaneous object-action detectors training in the videos is suggested to identify object-action pairs [52], which uses the two-stream faster R-CNN [53], and one fc layer operates on both streams' concatenated features. This approach is not just for human action recognition and includes actions, such as “cat eatings” or “dog jumping.” The attributes have also been used to understand human activities in an independent learning framework for recognizing objects and actions [54, 55]. The strong relationship between the objects and the actions is used for zero-shot recognition of action [56, 57].

HOI recognition through zero-shot learning is proposed in [13] that predicts the verb-object pairs from a still image. This method used a two-branch neural architecture that jointly trained for simultaneous recognition of objects and verbs. A similar approach is presented to zero-shot HOI recognition in video data [14]. An external knowledge graph is suggested [58] to validate predicted verb-object pairs and identify the most valid pairs. The external knowledge graph is made by extracting subject, verb, and object (SVO) triplets from knowledge bases [23, 59]. Each node in the graph is a verb or a noun (object), and its word embedding is the node's feature.

Our work is also scaling HOI recognition through zero-shot learning, but we focus on video data, which has more challenges. We present a neural architecture that can understand videos and detect objects and verbs in videos containing an HOI activity. We also proposed the use of side information to prevent predicting the invalid verb-object pairs (see Section 3.6).

### 2.3. Object Detection

Our proposed zero-shot learning method is compositional learning, in which the HOI decomposes into two components, verbs and objects. In other words, there are two components for recognition, verbs (human action) and objects. Recent advances in object detection have been achieved by the successful methods of region proposal [60] and region-based convolutional neural networks (R-CNN) [61]. Some works focused on processing time that is appropriate for real-time object recognition tasks. Only one processing step for recognizing the object in the image is suggested (YOLO) that concentrates on processing time [62]. Single-shot detector (SSD) [63] presented high-speed multiobject detection that uses different feature maps extracted from different layers of CNN to detect objects and their location in the image with varying sizes.

## 3. Proposed Approach

The primary purpose of this work is the ability to identify a novel HOI. We use the zero-shot learning approach because it increases identifiable HOIs without increasing HOI categories in training data. In other words, to train a recognizer model for a given number of classes, part of the target classes' data is sufficient. It is not necessary to have the data of all categories. Therefore, the need for training data is reduced. In this work, the input is a video (sequence of frames) containing a human-object interaction, and the output is a pair of “verb, object” as an HOI label.

Reducing the number of invalid predicted HOI classes, which are probably incorrect, is another goal of this work. For this purpose, the use of external information is suggested.

### 3.1. Zero-Shot on HOI Recognition

In zero-shot learning, the main class is decomposed into its components, and components recognition is applied instead of recognizing the main category. Identifying a new class in the zero-shot learning approaches is done by recognizing the class' components, which have been present separately in other classes seen by the model. In the test phase, the class components are recognized, and the predicted class is identified as a combination of the predicted components. Thus, a new combination of components, which the model did not see at the time of training, indicates the identification of a new class and is not labeling as a more similar existing class. Decomposing an HOI into a verb and object is previously introduced to identify the limited number of HOIs in still images [13]. Each HOI class decomposes into a verb and an object as its components. A particular verb can be performed on several different objects, for example, “writing on the whiteboard,” and “writing on the notebook.” Different verbs can also be performed on the same objects, such as “writing on the notebook” and “ reading a notebook.” If the system learns verb and object classes separately instead of HOI classes, it can recognize those verbs and objects in seen and unseen HOI classes and make verb-object pairs as an HOI class at test time. Suppose a particular object learned by a model from an HOI (with a specific verb) and that object exist in another HOI (with a different verb). In that case, the model can identify it, and it is not necessary to learn this object to model by second HOI class. The same applies to verbs. In other words, it is not required to feed all HOI categories to model for understanding all of them, and it only needs to have a training dataset, which includes all verbs and all objects. In other words, the problem of HOI recognition is decomposed into two recognition issues: verb recognition and object recognition. Therefore, the designed system must include two separate parts: verb recognition and object recognition.

Suppose the available HOI dataset includes ν verbs and ο objects. So, the identification system can recognize ν verbs and ο objects. Since an HOI class consists of a verb and an object, this system theoretically can identify |ν|.|ο| categories. Training a recognizer system for understanding |ν|.|ο| classes in a fully supervised manner needs to labeled training data for |ν|.|ο| HOI classes. But in the proposed approach, we only need labeled data for |ν| + |ο| categories. Also, since an HOI has one verb and one object, it can train both verb and object.

According to the above, the central system has two branches due to recognizing two components, namely, verb and object. The output of one branch is the predicted verb applied to the object, and the production of another branch is the object(s), which a verb is applied to it. The combination of the two outputs can be considered as a predicted HOI class.

The zero-shot learning methods have two stages: (1) predicting the components and (2) inferring the class label from predicted parts. The first stage in our problem is predicting the verb and objects, and the second is combining object and verb to infer HOI class. For the first stage, we use a two-branch structure that predicts the verb and objects. The second stage is done using side information to form an HOI class with verbs and objects obtained in the first stage.

The main idea of zero-shot on HOI recognition is introduced for the limited number of classes in still images [13]. Understanding video and, in particular, understanding HOI in video data is more challenging and more applicable than still image data, since, in this work, the zero-shot on HOI recognition in the video data is desired. Since the HOI is decomposed into two components (verb and object), the central recognizer system includes two main branches as two recognition tasks: one branch for verb recognition and one branch for object recognition. In this work, each recognition task is implemented by a neural structure.  Figure 1 shows the simple architecture for the mentioned system. The verb recognition branch uses the RGB frames and optical flow of input video, while the object recognition branch uses only RBG frames for detection. In each branch, the input video (RGB frames and/or optical flow) feeds to the CNN module for extracting high-level features, and then these features are used for the corresponding recognition tasks. The object recognition branch is more straightforward because it can be recognized from a single frame. So, we use a typical CNN-based object recognition structure. But the nature of verb recognition is more complicated than the object. To recognize the verb, we use a three-stream structure based on CNNs and RNNs.

### 3.2. Object Recognition Branch

Our focus and innovation are on the verb recognition branch. The object recognizer's desired output is the recognized objects from the input video and their reliability score. The objects of each frame of the input video are recognized by the existing successful object recognition method, SSD [63]. The SSD approach is based on the feed-forward CNN that produces a fixed-size collection of bounding boxes. After that, the score of object class instances in those boxes is predicted, and a nonmaximum suppression step makes the final detections. SSD is a fast object detection method because of eliminating bounding box proposals and subsequent feature resampling stage. The early network layers are based on standard architecture used for high-quality image classification. Some convolutional feature layers are added to the previous layers, which decrease in size progressively and allow predictions of detections at multiple scales. SSD uses separate predictors (filters) for different aspect-ratio detections. These filters apply to multiple feature maps to perform detection at multiple scales. So, the location of objects in an image and their reliability scores are predicted in a short time. See reference [63] for more details. In this work, we have not used the location information of the objects, and we have considered only the detected objects along with their score. Still, in future works, we can use the location information of the objects and salience areas of action to distinguish the target object from the background objects.

After detecting objects in each frame by SSD, the objects are obtained in the whole video. These objects combine with the recognized verb using side information (see Section 3.6) and reliability scores to make a valid verb-object pair, and the HOI class is identified.

### 3.3. Verb Recognition Branch

Verb recognition or, in general, activity understanding in video space is different from single image space. For activity-based video classification in deep learning approaches, usually, the features of each frame of input video extracted with a neural structure and class of video clip predicted by a set of features came from all frames. The use of two-stream structures is common for this purpose, in which one stream considers appearance cues (from RGB frames) and the other considers temporal cues (from optical flow). One input to activity understanding systems usually is a sequence of RGB frames of an input video clip. Much of an RGB image is the background and is not necessarily related to the activity. Hence, the features extracted from it are strongly affected by the background. Estimating susceptible areas to activity and extracting features from them can help us solve this problem. On the other hand, the background can also contain information about the event that occurred, and completely removing it can lead to performance degradation. Estimating the region related to activity and blurring the background can be useful. Thus, the RGB stream is split into two streams. The first stream estimates activity region patches and extracts features from them as patch-based representation. The second stream estimates the activity region, blurts other areas, and extracts features from the new RGB image as focal representation. The video data includes temporal information of what is happening, which is not in still images. The short-time temporal information can be represented by optical flow. Therefore, a common input to activity understanding systems can be an optical flow of input video for motion representation. These processing streams are described more detail in Section 3.5.

Given the above and that the nature of the verb's recognition is a subset of the action, we propose to use three inputs for the verb recognition task. These three inputs are estimated activity region patches, RGB image with blurred background, and the optical flow. So, the central system's verb recognition branch is a three-stream structure, including patch-based representation, focal representation, and motion representation. This three-stream structure was previously introduced for action recognition in the video [41]. We use this structure with a new feature aggregation technique to recognize the verb in the video.

### 3.4. Feature Aggregation

The final step in the recognition system is classification on a feature vector derived from three processing streams. Features obtained from each stream must aggregate to produce the final feature vector of each stream, and then the ultimate features of the overall system for classification are obtained. Conventional feature aggregation methods, such as average or max-pooling, represent the entire space of features as a single descriptor. These methods may be suboptimal to representing a video containing several subactions. Locally aggregation features were introduced in [64] and extended to spatiotemporal feature aggregation for action recognition as Action VLAD [7]. In this scenario, the features are clustered to K cluster and pooled jointly across space and time.  Figure 2 shows the difference between spatiotemporal and average or max-pooling aggregation. In the average and max pooling scenarios (Figures 2(a) and 2(b)), the entire space of the feature map is represented as a single descriptor. But in the Action VLAD scenario (Figure 2(c)), the feature space is represented by several (*K*) descriptors. With this technique, if the nature of the action consists of several sub-actions, we hope that it will be described more optimally. Therefore, it is more likely to recognize the correct action because the feature space is represented by multiple descriptors instead of one, and the deletion of information is less in the feature aggregation step.

Consider the extracted descriptors from each frame of the video in each spatial location be *x*_*i*.*t*_*ϵR*^*D*^, where *iε*{1 … *N*} is related to spatial location and *tε*{1 … *T*} is the frame index. For spatiotemporal aggregation, the descriptor space *R*^*D*^ is divided into *K* cells using *K* anchor points {*c*_*k*_} (stars in Figure 2(c)). Then, each descriptor *x*_*i*.*t*_ was assigned to one of the cells due to its distance from the anchor. The new descriptor is presented by the difference vectors calculated across the entire video as follows.

(1) $$\begin{array}{c} V\left[j,k\right]=\sum_{t=1}^{T}\sum_{i=1}^{N}\frac{e^{-\alpha {\left\|x_{i,t}-c_{k}\right\|}^{2}}}{\sum_{k{}^{\prime }}e^{-\alpha {\left\|x_{i,t}-c_{k^{\prime }}\right\|}^{2}}}\left(x_{it}\left[j\right]-c_{k}\left[j\right]\right), \end{array}$$

where *x*_*it*_[*j*] and *c*_*k*_[*j*] are the *j*-th component of the descriptor vector *x*_*i*,*t*_ and anchor *c*_*k*_. Parameter *α* is a tunable hyperparameter. The output is a matrix V where each column shows an aggregated descriptor related to one cell. The matrix intranormalized across columns, stacked, and L2-normalized [65] into a single descriptor of the entire video.

The difference vectors record the differences of extracted descriptors from subactions represented by anchors *c*_*k*_. So, this aggregating scenario can help to recognize the verbs that consist of some subactions.

### 3.5. Details of Each Stream in Verb Recognition

Our proposed model for verb recognition is a three-stream RNN-based structure. Each stream has three main processing steps, which are shown in Figure 3. The processing flow of the three streams is almost similar. Each stream's input is a sequence of frames in the form of RGB and/or optical flow. CNN extracts the convolutional features of each frame. Then, the extracted features of the *T* consecutive frames of video feed to LSTM blocks to represent the temporal information. The output is several spatiotemporal feature vectors. These vectors are then locally aggregated, and the final representation vector of each stream is prepared for the final classification. The following is a detailed description of each shown module in Figure 3.

#### 3.5.1. Path-Based Representation

This stream aims to find areas related to the target verb and use it to identify the verb. These regions are appropriate to represent the video clip based on the event that occurred in it.  Figure 4 shows the structure and processing process in this stream. The probable areas are selected using the method proposed by Papazoglou et al. [66], which uses the RGB frame and its optical flow. Other proposed regions are taken from the region proposal network (RPN) offered by Ren et al. [53]. The RPN extracts the areas that are prone to the presence of objects or entities. The RPN processes a still image and outputs lots of proposal windows, many of which are irrelevant. The final action patches were selected by merging the already and previously extracted regions. We see Algorithm 1 in [41] to choosing actionness patches process (see Algorithm 1 for more details). After selecting each frame's actionness patches, these are fed to CNN, and the convolutional features are extracted. All of these processes are related to the second block in Figure 3. After obtaining convolutional features of all *T* frames of the input clip, *T* feature vectors are fed to the RNN block and outputs *T* time-distributed feature vectors as the input video's temporal representation (third block in Figure 3). Of course, we use the LSTM block as an RNN for the video's temporal representation in all three streams. The final step in this stream is local feature aggregation (see Section 3.4). The time-distributed features are locally aggregated to the K descriptor, and the target activity is represented as its subactions. The output vectors are used to classify the occurred verb in the video clip, and the classification scores are predicted for each verb class.

#### 3.5.2. Focal Representation

As previously stated, much of an RGB image is the background and is not necessarily related to the event. So, it may lead to overfitting in the training phase if the background is not discarded. On the other hand, completely removing the background can lead to performance degradation because it can also contain information about the event. To handle this issue, after finding the foreground (selecting the probable area in patch-based representation stream), the background of the RGB image is blurred by a Gaussian low pass filter, and the other areas remain unchanged. The idea is inspired by the human focal vision system [41]. The resulting image is a focused image on the area prone to activity, which also retains background information. Subsequent steps, including convolutional feature extraction from all *T* frames, obtain time-distributed feature vectors using LSTM block, local feature aggregation, and predicting the classification scores, are quite similar to patch-based representation stream' steps.  Figure 5 shows the structure of this processing stream.

#### 3.5.3. Motion Representation

According to the contents of Section 3.3, the short-term temporal information in the video clip can be represented by optical flow. The RNN block can obtain long-term temporal information. So, the third stream of the verb recognition branch can be motion representation by optical flow (Figure 6). Each frame's convolutional features are extracted from optical flow by a CNN. The structure used for this stream is the motion-CNN proposed in [31]. The optical flow is computed between each consecutive frame using the Brox algorithm [67], which assumes the camera is static. As shown in Figure 6, the next steps are exactly like the two other streams.

As observed, the processing flow is the same in all three streams. Only the inputs of these streams are different. The first stream uses the salience patches of the input image, the second stream uses a focal image whose background is blurred, and the third stream uses optical flow. The output of each stream is classification scores for verb classes. Finally, these three streams' results are merged to recognize the target verb in the input video.

### 3.6. Side Information for Reducing Invalid HOIs

The zero-shot learning approach has two stages: (1) predicting the components and (2) inferring the class label from predicted parts. The first stage of this approach in our work is to recognize the verbs and objects done by the central system (two-branch HOI recognition system). The second stage is not complicated. It is enough to put the recognized verb and the object together and create the “verb-object” pair as a predicted HOI. But is any combination of verb-object acceptable? For example, the “eating a laptop” is a presumable verb-object combination that may be the central system's output. Is it acceptable? Of course not. So, there is a need for a scenario to solve this problem. We also tackle this problem in this work.

Many of our interactions with objects are based on our prior knowledge. We know that a s “laptop” is not edible, and we cannot eat it. Hence, we argue that the detected pair of verb-object (eating a laptop) is invalid. This argument is based on our prior knowledge. If the system has prior knowledge like humans, it can validate the output pairs and identify invalid states. In this case, the system realizes that “eating a laptop” is an incorrect HOI and seeks another verb or object to create a valid HOI.

The use of an external information graph is proposed for compositional learning for HOI [58]. The idea of using the side information comes from the concept of word embedding. The external graph encodes two essential types of knowledge: (1) the “affordance” of objects, such as “laptop can be held,” and (2) the semantic similarity between verbs or objects. SVO triplets define objects' affordance from the external knowledge base [59], and the similarity between verbs or objects is defined by lexical information from WordNet [68].

We propose a simple graph to modeling and using side information (Figure 7). The graph has three categories of nodes: verb, object, and interaction. Each verb and object is modeled as a separate node, and their attributes are provided from nltk [69] based on the concept of word embedding [70, 71]. These attributes are conceptual representations of words so that words with close meanings have similar attributes. For example, both the words “Sandwich” and “pizza” are related to a type of food, so they have a similar concept and are used in a similar sense. A verb node can only connect to an object node via a valid interaction node and create a graph path. So, each path in this graph shows a valid HOI. Valid HOIs are HOIs that exist in the dataset. There is no path between verbs together or objects together. Also, conceptually similar verbs (or objects) are connected with a link. The similarity between verbs (or objects) is computed by nltk [69]. The links help in finding the valid secondary HOIs. For example, let “hold a laptop” is a valid HOI (it existed in the database and its path exists in the graph), and “take a laptop” has not a path in the graph (it did not exist in the dataset), but there is a link within the “hold” and “take” nodes. Therefore, “take a laptop” can be a valid HOI (it is a valid secondary HOI). This rule also applies to object nodes.

The side information graph is used to validate the central system's results and enhance the overall performance. The central system's output is the classification score for the verb classes and the identified objects with their reliability score. The three verb classes with the highest classification score are combined with the identified objects to form possible “verb-objects ” pairs and are sorted by score. The validity of the obtained pairs is then checked using the side information graph, and the first valid pair is selected as the final predicted HOI class. In fact, this is the second stage of the zero-shot learning approach.

## 4. Results and Discussion

We present the results of our method in this section and compare it to some other works. The used dataset is introduced first, and then the implementation setups are described. Finally, we report our results and compare the proposed approach against state-of-the-art methods.

### 4.1. Dataset

For human action understanding in videos, several appropriate datasets have been provided and published, such as UCF101 [72], HMDB51 [73], and Actor-Action Dataset (A2D) [74]. Most of these datasets involve many human activities, not just HOIs. So, they are not suitable for the evaluation of HOI understanding tasks.

The recently published challengeable dataset for human activity understanding is Charades [12]. This dataset contains 9848 video clips of HOIs captured in real environments. It has 157 categories of human activities including some actions with “no interaction.s ” After excluding categories with “no interaction,s ” there are 149 valid HOI categories defined as verb-object pairs. This 149 category includes 34 verbs and 37 objects. Clips of this dataset cover both the third and first person's actions. We use the third person's clips of these 149 categories as our Charades benchmark.

We have two scenarios for evaluating our system. First, we assess the model for fully supervised HOI recognition and compare model performance with some state-of-the-art approaches. Afterward, we present the performance of the proposed model on the zero-shot detection of HOIs. For zero-shot analysis, we split each set of verbs and objects into two subsets. The object set is divided into subsets 1 and 2, and the verb set is divided into subsets A and B. So, we can provide four subgroups of HOI, including 1A, 1B, 2A, and 2B. For example, subgroup 1A consists of 49 HOIs whose verbs are in the verb subset A, and their objects are in the object subset 1. The same applies to the other three subgroups. Subgroup 1B includes 22 HOI classes, 2A includes 47 HOIs, and 2B includes 31 HOIs.

If we train the model with 1A + 2B, it does not see all HOIs but see all verbs and objects. So, it can identify the unseen HOIs that are in the subgroups of 1A and 2B. In other words, we are using 80 HOI classes (1A + 2B) to train a system that can recognize 149 HOI classes of the used dataset.

### 4.2. Implementation Details

The proposed system has three processing streams for verb recognition and one stream for object recognition. For the two spatial CNN streams of the verb recognition branch, an AlexNet architecture that pretrained on UCF sports, JHMDB, and HMDB51 datasets, is used. The first spatial network inputs are the action patches, and for the second spatial network, the proposed focal representation is fed. Moreover, a VGG16-RPN, which is trained on the ImageNet dataset, is used for region proposal to select the actionness patches process. For the 3rd stream of the verb branch as motion representation, we used the CNN network like the network architecture used by Gkioxari et al. [31]. This motion-CNN is pretrained on the optical flow images of UCF sports and JHMDB datasets. The optical flow is computed between each consecutive frame using the Brox algorithm [67]. For motion-CNN input, a 3D image is created by stacking the x-component, y-component, and optical flow magnitude. The FC7 layer of three CNNs extracts a 4096-dimensional feature vector for each input video frame. After obtaining feature vectors for all *T* frames of input clip in three CNNs, these feature vectors are fed to the RNN block and outputs *T* time-distributed feature vectors. For the RNN block, the LSTM module with 1024 hidden units is used. The last step before the final classification is local feature aggregation (see Section 3.4), in which the value 64 is selected for parameter *K*. The time-distributed features are locally aggregated with ActionVLAD, and the target activity is represented as its subactions. The output of this step is used to classify the occurred verb in the video clip. Two FC layers with the number of neurons equal to 256 and the number of verbs (here 34) are used as a classifier in each stream. For training the LSTM and its following dense network, a stochastic gradient descent optimizer (SGD) is utilized. The last FC layer determines the final prediction with a Softmax activation. For preventing overfitting, the flipping video frames technique is used for data augmentation. The learning rate is set to value 5 × 10^−5^. Also, we use *T* = 25 frames per video for both optical flow and RGB for learning and evaluation. The final verb class scores are obtained by averaging the three streams' results.

Another processing branch of the main system is the object recognizer. In this branch, the objects of each frame of input video are recognized by the existing successful object recognition method, SSD [63]. So, the objects are obtained in the whole input video. The results are objects with their reliability scores. These results combine with the recognized verb by using side information (see Section 3.5), and a valid verb-object pair is identified as the HOI class. Our deep learning system is implemented in python based on the Tensorflow open-source toolbox and Keras library.

### 4.3. Experimental Results

We start the experiments by comparing the zero-shot recognition accuracy of our initial model and the state of the art. The initial model has two spatial processing streams in the verb recognition branch (without motion representation).  Table 1 shows the results. The effect of using side information has also been investigated. The two last rows in Table 1 show the results of our simple system with or without side information (SI). The compared methods are all in the field of zero-shot learning, and, like us, they have tried to identify unseen classes. Our previous model [14] has one stream in verb branch recognition. The method [58] uses the convolutional graph networks, which learn how to compose classifiers for verb-noun pairs. The SES [68] and DEM [75] use the verb and noun embeddings, which are matched to visual features using L2 loss. CC [76] does not combine word embeddings but considers the composition of classifiers.

Our model better represents the video due to RNN blocks' use, which leads to better verb recognition. So, it has had better results. The use of side information graphs also had a positive effect on the results in Table 1. In Figure 8, two samples showed that they were misclassified without using the side information and were classified correctly after using the side information. The patterns of the right verbs and the false detected verbs are similar. Therefore, the model may classify incorrectly, but using the side information can correct such errors.

We propose using local feature aggregation to aggregate the feature maps extracted from input frames (Section 3.4). The proposed model for this evaluation is named 2Stream + WE + VLAD. The effect of this technique is shown in Table 2. The reported results indicate a slight performance improvement. We used the local aggregation after the RNN module, but it is possible to apply this technique to the outputs of the CNNs. The results show that its application to the RNN module has a slight performance improvement.

For the representation of the temporal information in the input video, the potential of recurrent neural networks (RNNs) has been exploited. Furthermore, the use of the optical flow of the input video as the 3^rd^ stream in the verb recognition branch has been investigated. The impact of using this stream is shown in Table 3. The model named **3Stream** **+** **WE** **+** **VLAD(rnn)** is our final proposed system, which uses the LSTM block as the RNN module. According to the results, using optical flow is observed in the slight improvement of system performance.

We used the RNNs for the representation of the temporal information in the input video. In previous evaluations, the LSTM block is used for the RNN module. Another choice is the GRU blocks, which are simpler than LSTMs and have a similar function. The GRU blocks are used with 1024 hidden units. The comparison between the use of the LSTMs and GRUs is made, taking into account the volume of training data. The results are shown in Tables 4–6. The values reported in Table 4 indicate that the GRU has a slight improvement to the LSTM. But looking at the results of Tables 5 and 6 shows the opposite. The difference is the amount of training data. In other words, the GRUs are simpler than the LSTMs, and they converge faster. So, we conclude that the GRU is appropriate for cases that the amount of training data is small (due to the rapid convergence), and the LSTM is the right choice for cases with a large amount of training data due to its excellent performance.

For the last evaluation, we examine our proposed system in a fully supervised scenario. In other words, the model sees all HOI classes in the training phase. 80% of all videos were used as training data, and the remaining 20% of videos were used for testing. Also, 10% of the training data are used as the validation set. We compared our model's performance to three other state-of-the-art action recognition methods on the Charades dataset. These three approaches are ActionVLAD [7], Sigurdsson et al. [8], and CoViAR [9], which are DNN-based. Our method in this evaluation for RGB input is 2Stream + WE + VLAD and for RGB + optical flow is 3Stream + WE + VLAD. According to the result of the previous evaluation, the LSTM has been selected for the RNN module. The results are reported in Table 7, which shows our method's better performance compared to the other three methods.

## 5. Discussion

This work's primary goal is to identify HOI classes that the model had not seen before. The main idea is to decompose the HOI into verb-object pairs and recognize them independently. Tables 1–3 compare our proposed system to the state of the art from the perspective of the intended purpose. Using the side information, representing the video by 3-stream structure and the RNN blocks, and using the local feature aggregation have ultimately led to our system's better performance. Using the side information has corrected some invalid misclassifications (see Figure 8.). Using the local feature aggregation technique leads to a better representation of some of the classes that consist of several subactions.

Figure 9 shows some misclassified samples of our final system. Observing these misclassified examples shows the visual patterns of the predicted classes are similar to the actual classes. These errors indicate that a lack of educational data for different categories has made the model unable to learn a general pattern. For example, the “opening” class has several patterns: opening the door, opening the refrigerator, opening the cabinet, and opening the laptop. If the model learns the pattern of “opening” for the class of opening the door, it can predict the “opening” in opening the cabinet without observing it during training. But the visual pattern of the “opening” of opening a laptop is different, and the model cannot predict correctly. If the training data for a verb exists in other cases, the model can learn a more general pattern and perform better during testing.

In addition to the zero-shot performance, which was the primary purpose of the work, we evaluate our method in a fully supervised scenario and compare it to some methods (Table 7). In this case, the model sees all HOI classes in the training phase. Our system's performance is slightly better due to its potential in video representation and the correction of some errors.

## 6. Conclusion

In this research, we propose a CNN-based system for HOI understanding in video data through a zero-shot learning approach, which can identify new classes that have not been seen before. So, the proposed method can identify more HOI classes than available HOIs for training and partly resolve data unavailability for all possible HOI classes. Our approach decomposes the HOIs to verbs and objects and addresses the problem as verb and object recognition in the videos. The model has a two-branch neural structure for two recognition tasks, and it uses a CNN for feature extraction. We showed that we could use 80 HOI classes (1A + 2B) to train a system that can recognize 149 HOI classes of the used dataset (1A + 2B + 2A + 1B). Of course, there can be more predictable classes in the real world because not all possible real-world combinations of objects and objects are in this used dataset. In other words, the information and potential of the available data can be better used.

We proposed using a local feature aggregation to better represent verbs (actions), especially verbs with multisubaction, before final classification. Conventional feature aggregation methods represent the entire space of features as a single descriptor, which may be suboptimal to representing a video containing several subactions. The used local feature aggregation technique prevents the deletion of information when merging features. So, the recognition of verbs with several subaction is improved.

We also proposed using side information to reduce the prediction of invalid verb-object combinations. Because of the separate recognition of verb and object, predicting the invalid verb-object pairs is possible. The side information shows the relations between verbs and objects defined by lexical information.

We showed the effect of each proposed technique on HOI recognition system performance. We also showed that our method could work slightly better than some fully supervised HOI recognition methods that reported the best results on the used dataset, although this improvement is tiny.

A more appropriate structure can be provided with better accuracy in recognizing the verb from the input video for future work. The distinction between background objects and activity-related objects can be used in future work, taking into account the location of the detected objects. We will also work on updating the system to learn new verbs or object classes without the need for data from previous classes. In other words, it is possible to apply incremental learning to the proposed system.

## Figures and Tables

**Figure 1:** A simple overview of the main system architecture. The verb recognition branch uses the RGB frames and optical flow of input video, while the object recognition branch uses only RBG frames for detection.

**Figure 2:** Difference pooling scenario for aggregate features. Different colors points correspond to different subactions in the video. (a) and (b) are good for similar features, but they do not adequately capture the complete distribution of features if the input video contains several subactions. Scenario (c) clusters features in spatiotemporal manner [59].

**Figure 3:** Block diagram of the process in each processing stream in the verb recognition branch shown in Figure 1. First, the convolutional features of each frame were extracted. Then, the whole input video is represented by the LSTM block. Finally, the elements are locally aggregated.

**Figure 4:** Patch-based representation. At first, the areas related to the target verb are detected, and the patches are extracted from the input frame. Then, the features of each patch in each frame are extracted. The LSTM block represents the whole input video. Finally, the elements are locally aggregated, and the class scores for each verb class are estimated.

**Figure 5:** Focal representation. At first, the area related to the foreground is detected from the input frame, and the background is blurred with a lowpass Gaussian filter. Then, the features of each blurred frame are extracted. The whole input video is represented by the LSTM block. Finally, the elements are locally aggregated and the class scores for each verb classes are estimated.

**Figure 6:** Motion representation. The short-term temporal information in the video clip can be represented by optical flow. In first, the features of each optical flow of each frame extracted. Then the whole input video is represented by the LSTM block. Finally, the elements are locally aggregated, and the class scores for each verb classes are estimated.

**Figure 7:** Side information graph. The green ellipse shows the verb nodes, the blue ellipse shows the object nodes, and the yellow ball shows an interaction. Each valid HOI is specified by the triple connected nodes (verb, interaction, and object). The conceptually similar verbs or objects nodes connected by a link (dashed lines).

**Figure 8:** Two samples were misclassified without using side information and were classified correctly after using the side information. In the first row, the true HOI class is “smiling at a book.“ Without using the side information, the predicted class was “playing, book.” After using the side information, the predicted class is “smiling, book.” In the second row, the true HOI class is “making a sandwich.s ” Without using the side information, the predicted class was “fixing, sandwich.” After using the side information, the predicted class is corrected as “making, sandwich.”

**Figure 9:** Such samples of incorrect classification of our final model. In the first row, the true class is “opening a laptop” but predicted as “fixing a laptop.” In the second row, the class of “fixing a vacuum” was predicted as “holding a vacuum.” Row 3 shows the “working at a table” that is predicted as “watching at a book,” and the final row shows the “grasping onto a doorknob,” which is predicted by our model as “fixing a door.”

**Table 1:** Zero-shot HOI recognition mAP on Charades dataset. The model trained with 1A + 2B and tested on 2A + 1B and all data.

Method	mAP (%) on the test set	
	All data	Unseen data (2A + 1B)
Chance	1.43	1.45
Compositional [58]	14.32	10.48
SES [68]	13.12	9.56
DEM [75]	11.78	8.97
CC [76]	14.31	10.13
1stream [14]	16.48	11.23
**2Stream – SI**	**17.8**	**14.83**
**2Stream** **+** **SI**	**19.5**	**16.08**

**Table 2:** The effect of local feature aggregation on HOI recognition performance. The model was trained with 1A + 2B and tested on 2A + 1B and all data.

Method	mAP (%)	
	ALL data	Unseen data (2A + 1B)
2Stream – WE - VLAD	17.8	14.83
2Stream + WE - VLAD	19.5	16.08
2Stream – WE + VLAD (rnn)	18.7	15.33
2Stream + WE + VLAD (rnn)	20.96	16.96
2Stream + WE + VLAD (cnn)	20.65	16.65

**Table 3:** The impact of the optical flow on the proposed system's performance. The model trained with 1A + 2B and tested on 2A + 1B and all data.

Method	mAP (%)	
	ALL data	Unseen data (2A + 1B)
2Stream – WE-VLAD	17.8	14.83
**3Stream – WE-VLAD**	**19.21**	**16.65**
2Stream + WE-VLAD	19.5	16.08
**3Stream** **+** **WE-VLAD**	**20.84**	**17.32**
2Stream + WE + VLAD (rnn)	20.86	16.96
**3Stream** **+** **WE** **+** **VLAD (rnn)**	**21.27**	**17.63**

**Table 4:** The impact of the RNNs (LSTM/GRU) on the proposed system's performance. Training and testing are performed on the same subset (averaged on four subsets).

Method	mAP (%)	
	LSTM	GRU
2Stream + WE - VLAD	20.28	20.33
3Stream + WE - VLAD	20.94	20.94
2Stream + WE + VLAD (rnn)	20.74	20.78
3Stream + WE + VLAD (rnn)	21.31	21.35

**Table 5:** The impact of the RNNs (LSTM/GRU) on the proposed system's performance. The model is trained with 1A + 2B and tested on all data.

Method	mAP (%)	
	LSTM	GRU
2Stream + WE - VLAD	19.5	19.42
3Stream + WE - VLAD	20.84	20.63
2Stream + WE + VLAD (rnn)	20.86	20.64
3Stream + WE + VLAD (rnn)	21.27	21.19

**Table 6:** The impact of the RNNs (LSTM/GRU) on the proposed system's performance. Training and testing are performed on all data.

Method	mAP (%)	
	LSTM	GRU
2Stream + WE - VLAD	22.45	22.20
3Stream + WE - VLAD	23.76	23.52
2Stream + WE + VLAD(rnn)	23.64	23.43
3Stream + WE + VLAD(rnn)	24.73	24.58

**Table 7:** HOIs recognition results (mAP(%)) on Charades dataset. The model sees all HOI classes in the training phase.

Method	mAP (%)	
	RGB	RGB + optical flow
ActionVLAD [7]	17.6	21.0
Sigurdsson et al. [8]	18.3	22.4
CoViAR [9]	21.9	24.1
**Ours**	**23.64**	**24.73**

## Data Availability

Previously reported image data were used to support this study and are available at https://doi.org/10.1007/978-3-319-46448-0_31. These prior studies (and datasets) are cited at relevant places within the text.
